The article "Study on Impact Mechanical Properties of Reentrant Bionic Automotive Energy Absorbing Box" was published in 2023. Journal: Appl Bionics Biomech.

# Study on Impact Mechanical Properties of Reentrant Bionic Automotive Energy Absorbing Box

**DOI:** 10.1155/2023/7283835

**Published:** 2023-01-05

**Authors:** Zhi-xin Liu, Wei-dong Liu

**Affiliations:** China Automotive Technology and Research Center Co. Ltd., Tianjin 300300, China

## Abstract

In order to impprove the protective effect of the automotive energy absorption (EA) box, the design of the reentrant bioinspired EA box is proposed, that is, novel bioinspired structures are inserted into the original EA box to improve the EA effect of the box. The improved bionic structures with curvature are designed according to the spider web: honeycomb structure (HS), arc-honeycomb structure (AHS), negative Poisson structure (PS), and arc negative Poisson structure (APS). A new bionic automobile energy absorbing box is constructed by combining with automobile energy absorbing box. Experiments and simulations further verify excellent mechanical properties of bionic structures. The results show that EA of AHS and APS is 117.2% and 105.8% of HS and PS. Their specific energy absorption is 112.2% and 102.7% of HS and PS. HS EA box structure, AHS energy absorption box structure, PS energy absorption box structure, and APS energy absorption box structure are 114.2%, 117%, 109.2%, and 116.2% higher than traditional EA box structures, respectively. The excellent characteristics of biological structures can provide ideas for structural design objectives of engineering applications and greatly simplify the process of optimal design.

## 1. Introduction

With the development of automotive energy absorption (EA) box, researchers have designed all kinds of novel optimization automotive EA box structures for various engineering fields [1–4]. Among all the existing automotive energy absorbing box designs, the protective energy absorbing characteristic is the most important. With the development of bionic optimization design, bionic automotive EA box design has gradually become a research focus [5–8].

In previous studies, researchers focused on EA [9], structural bearing capacity [10], and structural dynamic response [11] in the design of automotive EA box. In order to improve vehicle crash safety and reduce vehicle fuel consumption, Zhang et al. [12] took the wall thickness and geometric size of automotive EA box as design variables, combined with Latin hypercube experimental sampling technology, approximate model, and genetic algorithm, and optimized the design of automotive EA box under the conditions of strength, stiffness, and EA. Liang et al. [13] established a proxy model with box geometry parameters as independent variables and energy, acceleration, intrusion quantity, and mass as dependent variables. Multiobjective genetic algorithm is used to optimize the box structure, which provides a reasonable theoretical basis for the optimal design of the EA box. In view of the problems existing in energy-absorbing components in the process of low-velocity collision, Liu et al. [14] took the frontal impact test of low-velocity collision box as an example, analyzed the influence of various parameters on the model through mathematical analytical solutions and tests, and discussed the improvement method of the crash ability of collision box. It provides a useful method for further study of automobile. Pino et al. [15] discussed topological radial states in molecules with rotational symmetry and radial staggered jump amplitudes based on the explicit correlation between topological phase and the boundary state topological protector-edge correspondence. Wang et al. [16] introduced the structure of cactus into the design of EA box. By imitating the characteristics of cactus, they designed a corrugated angular structure with gradient distribution, which could effectively weaken the damage to the car body and improve the EA performance through stable folding deformation.

The article "Study on Impact Mechanical Properties of Reentrant Bionic Automotive Energy Absorbing Box" was published in 2023. Journal: Appl Bionics Biomech.

In this study, the design of the bioinspired EA box is proposed in order to improve the protective effect of the automotive EA box, that is, novel bioinspired structures are inserted into the original EA box to improve the EA effect of the box. The improved bionic structures with curvature are designed according to the spider web: honeycomb structure (HS), arc-honeycomb structure (AHS), negative Poisson structure (PS), and arc negative Poisson structure (APS). A new bionic automobile energy absorbing box is constructed by combining with automobile energy absorbing box. Experiments and simulations further verify excellent mechanical properties of bionic structures.

## 2. The Optimal Size Design of Bioinspired Structures

In nature, spider webs can withstand high-speed shocks without being destroyed, which means spider webs have excellent hardness, strength, and bending resistance. Also, spider webs, which are over trees several meters high, are at risk of falling or being hit by hard objects, but the web can withstand the impact and wrap the penguin's forehead around these objects, which means spider webs have excellent impact resistance and EA properties. To get bioinspired structures that have excellent functional characteristics of various parts of spider webs, the bioinspired design is implemented by mimicking the various parts of spider webs in this study [17–21]. According to the orderly arc arrangement of spider webs, two bioinspired structures are designed based on the optimal honeycomb and negative Poisson cell: HS, AHS, PS, and APS, as shown in Figure 1. The optimization design of bending radius and other parameters is carried out, as shown in Figure 2.

The article "Study on Impact Mechanical Properties of Reentrant Bionic Automotive Energy Absorbing Box" was published in 2023. Journal: Appl Bionics Biomech.

In this study, the HS and PS are fabricated using additive manufacturing FS3300PA machine. The material used in this experiment is nylon. However, in the process of three-dimensional (3D) printing bionic structure, different 3D printing parameters will affect the forming quality and mechanical properties of the structure. In order to meet the comparative requirements of structural impact resistance, the same additive manufacturing and printing parameters are used. 3D printing parameters such as volume forming rate (L/hr), scanning speed (m/s), cavity temperature (°F), laser power (W), and powder layer thickness (mm) are shown in Table 1.

The elastic modulus of nylon materials is *E*, *E* = 100 MPa, Poisson's ratio *υ*=0.39, and density *D* = 0.95 g/cm^3^. In order to ensure the accuracy of simulation calculations, #24 elastic–plastic material in LS-DYNA is selected for compression simulation calculation [22–24].

Bionic HS and PS have good impact resistance and EA performance, but bionic HS and PS have different EA and protection performance under different sizes. So, AHS and APS are changed by discrete variables, and the analysis results are shown in Figure 2.

It can be seen that with the addition of arcs in the HS and PS, the overall EA of the structure increases first and then decreases with the increase of the structural radius. When the radius is 3 mm, the HS and negative Poisson's ratio structure have the optimal characteristics, and the 3D HS and PS with the optimal radius are obtained.

## 3. Bionic Structure Analysis

### 3.1. Performance Indicators

To accurately measure protective performance of bioinspired structures, EA and specific energy absorption (SEA) are used in this paper [25–27].

EA is the total energy absorbed during compression, as shown in Equation (1)

(1) $$\begin{array}{c} EA=\int_{0}^{x_{0}}Fdx, \end{array}$$

where *x*_0_ is the compression distance, *F* is the compression force, and *x* is the compression displacement.

SEA is a great indicator of the energy absorbed, as shown in Equation (2). SEA is extremely vital within applications of protective engineering.

(2) $$\begin{array}{c} SEA=\frac{EA}{M}, \end{array}$$

where *M* is the mass of the bioinspired structure.

### 3.2. Mesh Adaptability Analysis

In the process of bionic structure compression, the size of the mesh size of the simulation structure can have a certain influence on the simulation results, so the adaptability analysis of the mesh size needs to be carried out [29]. Based on the basic bionic structural cell (HS, AHS, PS, APS), the convergence adaptability of the structural mesh size is analyzed under four different FEM mesh sizes of 0.5, 0.75, 1, and 1.5 mm by using LS-DYNA, as shown in Figure 3.

The article "Study on Impact Mechanical Properties of Reentrant Bionic Automotive Energy Absorbing Box" was published in 2023. Journal: Appl Bionics Biomech.

As shown in Figure 3, the EA of all bionic structural units is almost the same under the mesh sizes of 0.5, 0.75, and 1 mm. However, when the structural mesh size is 1.5 mm, there is contingency, and the EA is different. To improve the calculation convergence and the calculation speed, the structural mesh size of simulation analysis is set as 0.5–0.8 mm.

## 4. The Properties Analysis of Bionic Structures

To study EA and protection performance of HS and PS, compression simulations and experiments are used. The freedom of the structural bottom surface is constrained, that is, the models are placed in a fixed position and are compressed. To obtain accurate deformation and response effect, contact conditions are set for the simulation model. Auto surface contact is used for simulations. The friction coefficient between structures is set as 0.15. The compression direction of the structures is *y* direction, as shown in Figure 1. The deformation comparison of bioinspired structures is shown in Figure 4.

From the perspective of structural deformation, the bionic model with radian deforms uniformly in the compression process, while the traditional bionic structure will undergo hierarchical deformation after compression, which adversely affects the EA effect of the structure. Moreover, from the point of view of the stress cloud diagram, AHS and APS have uniform stress distribution, while the traditional bionic structure has uneven stress distribution in the compression process, resulting in stress concentration. This special regularity can be applied to structural design, and it can be preset to meet the engineering needs.

The mechanical properties' curves of bioinspired structures in quasi-static compression experiments and simulations' analysis are shown in Figure 5.

It can be seen from Figures 5(a) and 5(b) that the force–displacement curves of all structures are similar in shape. The force–displacement curve of the structure can be divided into three different stages: (1) elastic stage, (2) yield stage, and (3) platform stage. From the perspective of crashworthiness, AHS and APS have higher bearing capacity than those of HS and PS. The maximum force of HS, AHS, PS, and APS is 42.16, 50.96, 43.79, and 45.61 N, respectively. AHS and APS has the strongest EA, and their EA is 17.2% and 5.8% of HS and PS and their SEA is 12.2% and 2.7% of HS and PS. The excellent characteristics of biological structures can provide ideas for structural design objectives of engineering applications and greatly simplify the process of optimal design.

The article "Study on Impact Mechanical Properties of Reentrant Bionic Automotive Energy Absorbing Box" was published in 2023. Journal: Appl Bionics Biomech.

## 5. Impact Characteristics Analysis of Automotive Bionic Energy Absorbing Box

The car EA box is between the anticollision steel beam and the body rail. In the event of a collision, the EA box can collapse and absorb energy, so that part of the impact force can be absorbed, so as to protect the safety of the passengers in the car. In the event of a minor crash, the anticollision steel beam protects the body parts of the car, thus reducing the maintenance cost of the car owner. Furthermore, as a kind of metal thin-wall component, the EA box is prone to fold deformation during collision, which just meets the purpose of effectively absorbing collision energy and minimizing the damage of collision force to the longitudinal beam of the car body. However, the existing EA box is not satisfactory in terms of EA protection effect. In order to improve the protection effect of the EA box, the design of releasing EA box is proposed, that is, inserting a new releasing structure into the original EA box to improve the EA effect of the box. The specific design is shown in Figure 6.

Since the automobile collision occurred at a speed, the impact simulation is conducted on the bionic energy absorbing boxes at a speed of 4,000 mm/s, and the test results are shown in Figure 7.

The bionic EA boxes are deformed in a strong collision, which is mainly manifested as complete deformation, warping deformation, and fold deformation, among which the fold deformation is an ideal way of EA. From the perspective of deformation, the bionic EA box structure folds and deforms after collision, which has a good EA effect.

As shown in Figure 8(a), EA of the bionic automotive energy absorbing box is much higher than the traditional energy absorbing box structures. HS EA box structure, AHS EA box structure, PS EA box structure, and APS EA box structure are 14.2%, 17%, 9.2%, and 16.2% higher than traditional EA box structures, respectively. The one with new bionic structure is superior. It can be seen from Figure 8(b) that the bionic automotive EA box has higher mechanical bearing capacity and can play a better protective role. It has an extensive applicable degree, and structural radius design ideas can be also applied to the material microscopic design applications and it is of great research value.

## 6. Conclusion

In this paper, bioinspired structures are designed based on spider webs. The crashworthiness and EA properties of bioinspired structures are experimented and simulated. EA of AHS and APS is 117.2% and 105.8% of HS and PS. Their SEA is 112.2% and 102.7% of HS and PS. HS EA box structure, AHS EA box structure, PS EA box structure, and APS EA box structure are 14.2%, 17%, 9.2%, and 16.2% higher than traditional EA box structures, respectively. The excellent characteristics of biological structures can provide ideas for structural design objectives of engineering applications and greatly simplify the process of optimal design.

The article "Study on Impact Mechanical Properties of Reentrant Bionic Automotive Energy Absorbing Box" was published in 2023. Journal: Appl Bionics Biomech.

## Figures and Tables

**Figure 1:** Four bioinspired structures. (a) The spider web: (a_1_) the transverse shape of the honeycomb structure; (a_2_) the transverse shape of the negative Poisson structure. (b) Honeycomb structure. (c) Arc-honeycomb structure. (d) Negative Poisson structure. (e) Arc negative Poisson structure. *R* is the radius of the honeycomb structure. *r* is the radius of the negative Poisson structure.

**Figure 2:** Energy absorption analysis results of arc-honeycomb cell and arc negative Poisson cells with different radius of arc.

**Figure 3:** FEM convergence adaptability analysis of bionic structures.

**Figure 4:** The deformation and stress of bioinspired structures: (a_1_–a_4_) HS stress distribution diagrams at compression strain of 0.044, 0.105, 0.204, and 0.245; (b_1_–b_4_) AHS stress distribution diagrams at compression strain of 0.044, 0.105, 0.204, and 0.245; (c_1_–c_4_) PS stress distribution diagrams at compression strain of 0.044, 0.105, 0.204, and 0.245; (d_1_–d_4_) APS stress distribution diagrams at compression strain of 0.044, 0.105, 0.204, and 0.245.

**Figure 5:** The mechanical characteristic curves of bionic structures: (a) the experiment and simulation force–displacement curves of honeycomb structures; (b) the experiment and simulation force–displacement curves of negative Poisson structures; (c) EA histogram of bionic structures; (d) SEA histogram of bionic structures.

**Figure 6:** Bionic structure design of automotive energy absorbing box: (a) the HS automotive energy absorption box; (b) AHS automotive energy absorption box; (c) PS automotive energy absorption box; (d) APS automotive energy absorption box; (e) the automotive energy absorption box; (f) the right view of the automotive energy absorption box; (g) the front view of the automotive energy absorption box; (h) the vertical view of the automotive energy absorption box. In order to better compare the effect, steel is used in the simulation of bionic automobile energy absorption box [28].

**Figure 7:** The deformation and stress of automotive energy absorbing box: (a_1_–a_3_) HS automotive energy absorbing box stress distribution diagrams at compression strain of 0.105, 0.204, and 0.285; (b_1_–b_3_) AHS automotive energy absorbing box stress distribution diagrams at compression strain of 0.105, 0.204, and 0.285; (c_1_–c_3_) PS automotive energy absorbing box stress distribution diagrams at compression strain of 0.105, 0.204, and 0.285; (d_1_–d_3_) APS automotive energy absorbing box stress distribution diagrams at compression strain of 0.105, 0.204, and 0.285; (e_1_–e_3_) the automotive energy absorbing box stress distribution diagrams at compression strain of 0.105, 0.204, and 0.285.

The article "Study on Impact Mechanical Properties of Reentrant Bionic Automotive Energy Absorbing Box" was published in 2023. Journal: Appl Bionics Biomech.

**Figure 8:** The mechanical characteristic of bionic automotive energy absorbing box structures: (a) the EA histogram of bionic automotive energy absorbing box structures; (b) the simulation force–displacement curves of bionic automotive energy absorbing box structures.

**Table 1:** 3D printing parameters.

Parameters	Volume forming rate (L/hr)	Scanning speed (m/s)	Build cavity temperature (°F)	Laser power (W)	Powder layer thickness (mm)
Tensile sample	76	7.8	6,400	31	0.1

## Data Availability

The data and materials that support the findings of this study are available from the corresponding author upon reasonable request.

## References

[1] Zhang X., Zhao X. Research on structure optimization of automobile energy absorbing box based on collision safety.

[2] Zhuang W., Shi H., Xie D., Chen Y., Yang C. (2019). Research on the lightweight design of body-side structure based on crashworthiness requirements. *Journal of Shanghai Jiaotong University (Science)*.

[3] Uma Devi B., Vamsi Krishna C., Mohan Swaroop P. (2014). Design simulation of crash box in car. *International Journal of Engineering Research & Technology (IJERT)*.

[4] Koike A., Yokoyama A., Akita R., Sukegawa Y., Kawamura K., Oohira H. Development of the high performance FRP crush box: a report of JSAE FRP working group activity. Analysis of collapse mechanism of the trigger part of FRP crush box.

[5] Li Q.-F., Liu Y.-J., Wang H.-D., Yan S.-Y. Finite element analysis and shape optimization of automotive crash-box subjected to low velocity impact.

[6] Chaochao L. I., Xiang J., Wang H. (2017). The influences of structural parameters of energy-absorbing box for automobile bumper on the energy absorption characteristics during low speed collision. *Journal of Xi’an Jiaotong University*.

[7] Yu Y., Guo Y., Fei L., Wang S., Huang X. (2017). Structure design and crashworthiness analysis of aluminum alloy energy-absorbing box. *Automobile Applied Technology*.

[8] Liu Y. J., Xia C. Y., Ding L., Liu C. H. (2013). Influence of material on automotive crash-box crashworthiness subjected to low velocity impact. *Advanced Materials Research*.

[9] Yusof N. S. B., Sapuan S. M., Sultan M. T. H., Jawaid M., Maleque M. A. (2017). Design and materials development of automotive crash box: a review. *Ciência & Tecnologia dos Materiais*.

The article "Study on Impact Mechanical Properties of Reentrant Bionic Automotive Energy Absorbing Box" was published in 2023. Journal: Appl Bionics Biomech.

[10] Li Y. T., Wang H. (2021). The influence of rapid prototyping technology on optimization of automobile energy-absorbing box. *Key Engineering Materials*.

[11] Song K., Yang B. C. (2014). Collision simulation and analysis of energy-absorbing box for vehicle. *Applied Mechanics and Materials*.

[12] Zhang Q., Zhao L., Zhang Q., Wei X. Geometry parameter optimization method for automobile energy-absorbing box.

[13] Liang J. S., Shi G. Y., Luo M. B. (2016). Structure optimization design of energy-absorbing box for automobile. *Machinery Design & Manufacture*.

[14] Liu Y., Ding L., Yan S., Yang Y. (2009). Computer simulations and experimental study on crash box of automobile in low speed collision. *Proceedings of SPIE*.

[15] Pino J. P., Alves P., Gouveia J. D., Marques A. M., Dias R. G. (2020). Topologically protected states in a spider web lattice. *Physical Review Research*.

[16] Wang C. Y., Lu G. C., Zhao W. Z., Wang Y. (2020). Modeling and multi-objective optimization of a bionic crash box with folding deformation. *Structural and Multidisciplinary Optimization*.

[17] Chu X. J. (2011). Test study on bionic technology of anti-scouring protection for subsea pipelines. *Equipment Manufacturing Technology*.

[18] Guo X., Dong X., Yu Z. (2020). Study on the mechanical properties of bionic protection and self-recovery structures. *Materials*.

[19] Jun-Jie L. I., Hou Z. M., Tian P. S. (2017). Bionic grass protection technology for submarine pipelines under the threat of huge wave erosion. *Coastal Engineering*.

[20] Yao G., Liu R., Xu Z. (2021). Study on quasi-static mechanical properties of four 3D-printed bio-inspired structures based on functional relationship. *Composite Structures*.

[21] Sun R. J., Gu S. C., Xie X. B., Gao K., Zhang Y. Z. (2018). Research on bionic impact compacting bits. *Coal Geology & Exploration*.

[22] Zhang W., Li D., Zhu J. (2021). A landing impact simulation test method for lunar lander. *Journal of Physics: Conference Series*.

[23] Wang H., Zhou C., Zhao C., Ren J., Zhong J. (2020). Structural design and impact simulation of glass fiber fragile cover of rocket. *Journal of Physics: Conference Series*.

[24] Goyal C., Kumari D., Bhat G. A. WITHDRAWN: Numeric projectile impact simulation on a server utilizing LS-DYNA. *Materials Today: Proceedings*.

[25] Jishi H. Z., Alia R. A., Cantwell W. J. (2022). The energy-absorbing characteristics of tubular sandwich structures. *Journal of Sandwich Structures & Materials*.

[26] Zhu G., Zhao Z., Hu P., Luo G., Zhao X., Yu Q. (2021). On energy-absorbing mechanisms and structural crashworthiness of laterally crushed thin-walled structures filled with aluminum foam and CFRP skeleton. *Thin-Walled Structures*.

The article "Study on Impact Mechanical Properties of Reentrant Bionic Automotive Energy Absorbing Box" was published in 2023. Journal: Appl Bionics Biomech.

[27] Rogala M., Gajewski J., Ferdynus M. (2020). The effect of geometrical non-linearity on the crashworthiness of thin-walled conical energy-absorbers. *Materials*.

[28] Achitei D. C., Abdullah M. M. A. B., Minciună M. G., Perju M. C. (2017). Study on characteristics modification of rul 1 steel. *European Journal of Materials Science and Engineering*.

[29] Liu R., Yao G., Xu Z. (2022). Study on functional mechanical performance of honeycomb array structures inspired by gideon beetle. *Journal of Bionic Engineering*.

